# Beta-mangostin demonstrates apoptogenesis in murine leukaemia (WEHI-3) cells in vitro and in vivo

**DOI:** 10.1186/s12906-017-1867-0

**Published:** 2017-07-17

**Authors:** Fatima Abdelmutaal Ahmed Omer, Najihah Mohd Hashim, Mohamed Yousif Ibrahim, Abdulmannan F. Aldoubi, Pouya Hassandarvish, Firouzeh Dehghan, Noraziah Nordin, Hamed Karimian, Landa Zeenelabdin Ali Salim, Mahmood Ameen Abdulla, Karim Al-Jashamy, Syam Mohan

**Affiliations:** 1 Department of Pharmacy, Faculty of Medicine, University of Malaya, 50603 Kuala Lumpur, Malaysia; 2 Center for Natural Product Research & Drug Discovery, University of Malaya, 50603 Kuala Lumpur, Malaysia; 3 Department of pharmacology , Faculty of Medicine, University of Malaya, 50603 Kuala Lumpur, Malaysia; 4 Tropical Infectious Diseases Research and Education Center, Department of Medical Microbiology, Faculty of Medicine, University of Malaya, 50603 Kuala Lumpur, Malaysia; 5 Department of Exercise Science, Sports Center, University of Malaya, 50603 Kuala Lumpur, Malaysia; 6 Medical Science 1, Faculty of Medicine and Health Sciences, Universiti Sains Islam Malaysia, 55100 Kuala Lumpur, Malaysia; 7 Department of Biomedical Science, Faculty of Medicine, University of Malaya, 50603 Kuala Lumpur, Malaysia; 8 Medical School, SEGi University College, 47810 Petaling Jaya, Selangor Malaysia; 9 Medical Research Centre, Jazan University, Jazan, 11420 Saudi Arabia

**Keywords:** Beta-mangostin, Leukaemia, Apoptosis, WEHI-3 cell line, BALB/c mice

## Abstract

**Background:**

Beta-mangostin (BM) is a xanthone-type of natural compound isolated from *Cratoxylum arborescens.* This study aimed to examine the apoptosis mechanisms induced by BM in a murine monomyelocytic cell line (WEHI-3) in vitro and in vivo*.*

**Methods:**

A WEHI-3 cell line was used to evaluate the cytotoxicity of BM by MTT. AO/PI and Hoechst 33342 dyes, Annexin V, multiparametric cytotoxicity 3 by high content screening (HCS); cell cycle tests were used to estimate the features of apoptosis and BM effects. Caspase 3 and 9 activities, ROS, western blot for Bcl2, and Bax were detected to study the mechanism of apoptosis. BALB/c mice injected with WEHI-3 cells were used to assess the apoptotic effect of BM in vivo.

**Results:**

BM suppressed the growth of WEHI-3 cells at an IC_50_value of 14 ± 3 μg/mL in 24 h. The ROS production was increased inside the cells in the treated doses. Both caspases (9 and 3) were activated in treating WEHI-3 cells at 24, 48 and 72 h. Different signs of apoptosis were detected, such as cell membrane blebbing, DNA segmentation and changes in the asymmetry of the cell membrane. Another action by which BM could inhibit WEHI-3 cells is to restrain the cell cycle at the G1/G0 phase. In the in vivo study, BM reduced the destructive effects of leukaemia on the spleen and liver by inducing apoptosis in leukaemic cells.

**Conclusion:**

BM exerts anti-leukaemic properties in vitro and in vivo*.*

## Background

Leukaemia, or blood cancer, is a dangerous widespread global affliction characterized by the overproduction of abnormal white blood cells in the bone marrow [1]. According to World Health Organization (WHO), the incidence of leukaemia is estimated at 2.5 per 100,000 individuals in Asian countries [2]. The causes of leukaemia are attributed to inherited and environmental (non-inherited) factors, such as smoking, ionising radiation, chemicals (benzene), chemotherapy, and Down syndrome [3].

Nowadays, the cure of leukaemia is a multidisciplinary effort that includes haematopoietic stem cell transplantation, radiotherapy, and chemotherapy; however, these approaches are not completely satisfactory [4]. Many studies have concentrated on discovering new therapeutic agents, particularly from medicinal plants that impede the progress of malignant cells [5]. The most efficient approach for the suppression of malignant cells is to induce apoptosis, which is a highly regulated process of programmed cell death. Apoptosis plays an essential physiological role in providing an effective way to remove redundant or damaged cells from tissues, thereby securing tissue homeostasis [4].

*Cratoxylum arborescens* is an Asian medicinal plant belonging to the Guttiferae family and is used traditionally as a therapy for fever, coughs, diarrhoea, itches, ulcers, and some abdominal disorders [6]. Phytochemical analysis of this plant has shown the presence of xanthones compounds [6]. Beta-mangostin (BM) (Fig. 1) is one of the major constituents of *C. arborescens*.

**Fig. 1:** **a** The chemical structure of beta-mangostin. **b** The IC_50_ concentration of BM against WEHI-3 in 24 h

Recent studies from our laboratory revealed that BM has a potential anticancer effect against breast cancer [7, 8].

The murine WEHI-3 leukaemia cell line was first established in 1969 and showed characteristics of myelomonocytic leukaemia. This cell line has been used to induce leukaemia in BALB/c mice in order to assess the anti-leukaemic effects of agents [9]. The present study was performed to investigate these anti-leukaemic effects, as well as the mechanism of action of BM on WEHI-3 leukaemic cells in vitro and in vivo.

## Methods

### Chemicals and materials

Fetal bovine serum albumin (FBS), RPMI 1640 media, penicillin–streptomycin, trypsin-EDTA 10X, and ribonuclease A (RNase A) were purchased from Nacalai Tesque, Japan, while dimethylsulphoxide (DMSO) (Merck Co, Germany), 3-(4, 5-dimethylthiazol-2-yl)-2, 5-diphenyltetrazolium bromide MTT, phosphate buffered saline (PBS), propidium iodide (PI), and acridine orange (AO) were purchased from Macalai, Japan. An Annexin V-FITC Apoptosis Detection Kit (APO Alert Annexin V) was obtained from Clean Tech, California, USA. Caspases 3&9 Colorimetric Assay Kits from R&D Systems, BD Pharmingen. The antibodies used for western blot, Bax, Bcl2, and B-actin and secondary antibodies (Goat pAb to Rb IgG) were obtained from Abcam, Inc. (California, USA) Multiparameter Cytotoxicity 3 Kit (Thermo Scientific, PA, USA).

### Cell line

A murine myelomonocytic cell line (WEHI-3) was obtained from the American Type Culture Collection (ATCC), then sub-cultured in a tissue culture flask measuring 75 cm with RPMI 1640 media mixed with 10% of bovine serum albumin and 1% penicillin-streptomycin; this was kept in an incubator at 5% of CO_2_ saturation at a temperature of 37 °C.

### Plant and compound isolation

The collection of the *C. arborescens* plant for the extraction, isolation, and identification of BM as a pure compound has been reported in detail in a study by one of our group [7].

### Cytotoxic effects of BM on WEHI-3

This assay was performed to evaluate the cytotoxicity of BM with the purity (99%) determined by HPLC-LC 20 AD (Shimadzu, Japan) [10] on WEHI-3. Briefly, 5 × 10^3^ cells/mL of WEHI-3 leukaemic cells were seeded per well in 96-well plates; these cells were treated with BM (dissolved in 1% DMSO) at different concentrations (100, 50, 25, 12.5, 6.3, 3.5, 1.5, and 0 μg/mL), and then incubated at 37 °C with 5% CO^2^ saturation for 24, 48 and 72 h. After incubation, 20 μL of MTT solution (5 mg/mL) was added to each well, followed by 4 h of incubation. Next, 100 μL of DMSO was then added to each well to dissolve the formazan crystals, and the density was measured using an ELISA microplate reader (Tecan Group Ltd., Männedorf, Switzerland) at 570 nm. The inhibition of BM of cell growth was expressed as an IC_50_ value.

### Quantification of apoptosis using propidium iodide and acridine orange double staining

WEHI-3 cells were seeded at a concentration of 2 × 10^5^ cells/mL in a 25-mL culture flask. They were then treated with IC_50_ concentration (14 μg/mL) of BM for 24, 48 and 72 h; the cells were kept in 5% CO_2_ at 37 °C, then collected and centrifuged at 1500 rpm. The supernatant was discarded, and the cell pellet was washed twice with cold PBS. Up to 10 μL of a mixture of the fluorescent dyes AO (10 μg/mL) and PI (10 μg/mL) was added to the pellet for cell resuspension. The stained cell suspension was placed on a glass slide and covered with a cover slip. Before the dye fluorescence faded, the slides were examined for 30 min under a UV-fluorescence microscope (Leica attached with Q-Floro software) in accordance with standard procedures. Viable cells appeared with a green nucleus and an intact structure, whereas early apoptotic cells exhibited a bright green nucleus showing condensation of the nuclear chromatin. Late apoptotic cells displayed dense orange areas of chromatin condensation.

### Hoechst 33342 staining

For the further detection of apoptosis signs induced by BM, bisbenzimidazole (Hoechst 33342) stain was used to reveal chromatin condensation, which is one of the hallmarks of apoptosis. Afterwards, the WEHI-3 cells were treated for 24, 48 and 72 h at 14 μg/mL. Both treated and control leukaemic cells were collected and centrifuged at 1500 rpm, and the pellet was washed twice with cold PBS, then centrifuged. Hoechst dye (10 μg/mL) was subsequently added. Stained cells were suspended and placed on a slide, covered with a cover slip, and examined under a UV-fluorescence microscope (Leica attached with Q-Floro software).

### Annexin V assay

WEHI-3 (5 × 10^3^ cells/mL) were treated with 14 μg/mL of BM and incubated for 24, 48 and 72 h, and then the cells were collected and centrifuged at 1500 rpm. The pellet was resuspended in 1X binding buffer and incubated for 1 h. Afterwards, Annexin V (5 μL) and PI (10 μL) were added. The cells were kept in the dark at room temperature for 15 min. Samples were run and analysed by FACS Canto II cytometry (BD Biosciences, San Jose, CA, USA).

### Determination of reactive oxygen species production

The capability of BM to produce reactive oxygen species (ROS) was evaluated using 2′,7′-dichlorofluorescin diacetate (DCFH-DA). WEHI-3 cells (5 × 10^3^ cells/mL) were seeded in each well of black 96 wells. Then, cells were treated with specific doses of BM. After an incubation period of 24 h, DCFH-DA (100 μL) was added, and the suspensions were incubated for 30 min at 37 °C. The fluorescence was measured at 485-nm via a fluorescence microplate reader (Tecan Infinite M 200 PRO, Männedorf, Switzerland).

### Multiple cytotoxicity assays

Multiple cytotoxicity assays were run to determine the involvement of mitochondria in the apoptosis process induced by BM. WEHI-3 cells were seeded in the black 96 well plate at 5 × 10^3^ cells for each well, followed by treatment with BM at 14 μg/mL; the plate was incubated at 37 °C for 24, 48h. According to the protocol, several solutions were added to each well, including 50 μL of live cell staining, 100 μL of fixation solution, 100 μL of 1X permeabilization, and 100 μL of 1X blocking buffer for 30, 20, 10, and 15 min incubation, respectively. After each step, prior to exchanging the solution, a total of 100 μL of 1X wash buffer was added to each well for washing. Afterward, each well was washed with 1X wash buffer, and 50 μL of the primary antibody solution was added.

The plate was incubated for 1 h in a dark area at room temperature. The secondary antibody (50 μL) was added after removing the primary antibody and incubated for 1 h. Then, the cells were washed three times with 1X wash buffer. The ArrayScan HCS Reader was used to read the plate.

### Activities of caspases 3/7, 9

Caspases are intracellular protease enzymes involved in apoptosis. To assess the susceptibility of BM to stimulate the enzymatic activity of caspases 3/7 and 9 the WEHI-3 cells were treated for 24, 48 and 72 h. Then, cells were centrifuged at 1500 rpm for 5 min, the pellet was washed in cold PBS and mixed with 25 μL of manufactured lysis buffer, and then incubated on ice for 10 min. Then, the mixture was centrifuged at 10,000×*g* for 1 min, and the supernatant was collected and transferred to 96-well plates. After that, 50 μL of reaction buffer and 5 μL of the substrate for caspase-9 (LEHD-PNA) and caspase-3(DEVD-PNA) were added. The plates were incubated at 37 °C for 2 h and were then read by a Tecan Infinite®200 Pro microplate reader (Tecan, Männedorf, Switzerland) at a wavelength of 405 nm.

### Western blot

Apoptosis is a biochemical event leading to characteristic cell changes (morphology) and death. This event is controlled by several proteins classified as anti-apoptotic proteins, such as Bcl2, and apoptotic proteins, such as Bax. To study the effect of BM on these two proteins, WEHI-3 cells were cultured in 75 mL flasks, then treated with BM at 14 μg/mL for 24, 48 and 72 h.

Subsequently, after the incubation times, the PRO-PREPTM (iNtRON, Biotechnology, Korea) kit was used to extract the whole proteins, and the Bio-Rad kit was employed for protein quantification. Approximately 10–14% of sodium dodecylsulphate polyacrylamide gel electrophoresis (SDS-PAGE) was used to run the samples for 2 h to obtain separated bands of targeting proteins; afterwards, the bands were transferred from the gel to a polyvinylidene fluoride (PVDF) membrane (Bio-Rad). The membrane was washed with distilled water, and BSA was used to block the membrane for 60 min. Each primary antibody for targeting proteins was diluted 1:1000 and incubated with the membrane overnight, before being washed with Tween 20 PBS (TPBS). The membrane was incubated for 1 h with a suitable secondary antibody 1:2000. To visualise the protein bands on the membrane, a colorimetric horseradish peroxidase (HRP) substrate, 4-chloro-1-naphthol (4CN) (Bio-Rad) kit was used. To capture images of the membrane, a UV gel documentation system (Biospectrum 410, UVP) was used.

### Cell cycle analysis

To determine at which phase BM can arrest the cell cycle of the treated and untreated leukaemic cells, (5 × 10^3^ cells/ml) of WEHI-3 cells were harvested and centrifuged at 1800 rpm for 5 min. The pellet was washed twice with pre-warmed PBS (37 °C) and then centrifuged. Subsequently, 700 μL of 90% cold ethanol was added, and the mixture was kept overnight at 4 °C. After incubation, the cell suspension was centrifuged at 1800 rpm for 5 min, and the ethanol was discarded. The cell suspension was then washed with PBS, and 700 μL of pre-warmed PBS was added to the pellet and mixed; this was followed by the addition of 25 μL of RNase (10 mg/mL) and 50 μL of PI (1 mg/mL) prior to incubation for 1 h, respectively. The sample was run and analysed by FACS Canto II cytometry (BD Biosciences, San Jose, CA, USA).

### Animals used in the in vivo study

The acute toxicity effect of BM was studied in mice (500 mg/kg) by Suvitha Syam in 2014, who reported it as a safe compound [10]. BALB/c is a type of laboratory mouse useful for research in cancer and immunology [11]. The murine monomyelocytic WEHI-3 leukaemia cell line was established from this mouse; consequently, BALB/c provides an ideal model of myelomonocytic leukaemia to use when studying the effects of potential therapeutic drugs on WEHI-3. To achieve one of the current research objectives in estimation of the anti-leukaemic property of BM under physiological conditions, WEHI-3 cells were injected intraperitoneally into the BALB/c mice.

Sixty male BALB/c mice, aged 8 weeks and weighing 22-25 g, were obtained from the Laboratory Animal Centre, University Putra Malaysia, and kept for 15 days in the Animal Centre of the University of Malaya before the experiment started at 25 ± 3 °C and relative humidity 55–60 °C (a cycle of 12 h–light and 12 h–dark). This study was approved by the Institutional Animal Care and Use Committee, University of Malaya (UM IACUC), under ethics number FAR/2310512013/FAAO (R).

### Leukaemia inoculation in BALB/c mice and experimental design

The aim of this study was to assess the effect of BM on monomyelocytic WEHI-3 leukaemia cells in the biological system of the BALB/c mice; the in vivo study was designed to achieve this aim.

In this experiment, 60 male BALB/C mice were used. They were divided into six groups (0–6), with each containing 10 mice. Group 0 was comprised of healthy controls (not injected with WEHI-3, leukaemic cells); whereas the other five groups (1–5) were injected intraperitoneally (i.p) with WEHI-3 cells (1 × 10^6^ cells/mice) [12] using a 1 ml syringe with a 27G needle. Then, 4 days after the inoculation, the mouse blood smear was performed to confirm the induction of leukaemia; following that, the leukaemic mouse group 1 was untreated (Leu), group 2 was treated daily with Tween 20 (the vehicle) (Leu + Tween 20), and groups 3 and 4 were treated with BM 30 mg/kg(Leu + BM-LD) and 60 mg/kg (Leu + BM-HD), respectively. These doses were dissolved in 200 μL of Tween 20, then taken orally (gavage) and daily, for 3 weeks [13], [14]. Vinblastine was used as a positive control (120 μg/kg) [15]. This experiment was carried out in the Animal Centre of the University of Malaya for 21 days. During this time, all the mice in the different groups were fed and supplied with water normally, and body weight was measured every 4days. At the end, the mice from all the groups were sacrificed and their livers and spleens were collected, weighed, and stored for histopathological and terminal deoxynucleotidyl transferase dUTP nick end-labelling (TUNEL), assays.

### Haematoxylin–eosin staining and histopathology

The mouse spleens and livers of all groups were collected, fixed in a 10% formalin solution, and embedded in paraffin in the blocks. Sections of 5 μm were stained with haematoxylin–eosin (H&E). The histology of the stained tissues was identified by a pathologist under a microscope.

### TUNEL assay

To detect apoptotic cells in the spleen and liver, the TUNEL assay (Promega, USA) was performed following the manufacturer’s instructions. The slides were deparaffinised by immersing them in clean xylene. Secondly, the tissues were rehydrated via immersion for 3 min in 100, 95, 85, 70, and 50% of ethanol, sequentially, and 0.85% NaCl was used to wash the slides. Then, the tissue was immersed in PBS and 4% methanol-free aldehyde for 15 min, respectively. The tissue was covered by 100 μL of proteinase K solution (20 mg/mL), and 100 μL of equilibration buffer was used to overlay the tissue after washing with 4% methanol–free aldehyde and PBS. This was followed by the addition of 50 mL of rTdT buffer incubated in a dark area for 1 h. At the end of this step, the slides were immersed in a sodium citrate solution for 15 min. The excess Florescent-12-dUTP was washed with PBS. Then, the tissues were stained with PI solution (1 μg/mL in PBS) for 15 min, before being covered with coverslips. A fluorescence microscope was used to observe any changes.

### Statistical analysis

Data were expressed as mean ± SD, and one-way ANOVA was used to evaluate the differences between groups. Values of * *p* < 0.05 were considered statistically significant. GraphPad Prism 5.0 was used to present the data.

## Results

### BM repressed the WEHI-3 cell viability

The MTT assay was implemented to measure the cytotoxic efficacy of BM towards WEHI-3 cells. As described in Fig. 1, BM significantly inhibited the growth of WEHI-3 cells after 24 h at 14 μg/mL.

### Acridine Orange – Propidium Iodide double staining cell morphological analysis

Observation of the WEHI-3 treated cells by BM under a fluorescence microscope after 24 h showed morphological changes related to early apoptosis, in which treated cells appeared with a bright green colour. Treatment of the cells with BM at 48 and 72 h revealed morphological alterations related to late apoptosis; treated cells were seen to have a reddish-orange colour. Furthermore, the number of apoptotic cells increased in a time-dependent manner compared to untreated cells, indicating that BM had induced apoptosis in WEHI-3 cells (Fig. 2).

**Fig. 2:** Fluorescent photomicrograph of AO/PI double-stained WEHI-3cells. The cells were treated with BM at 14 μg/mL for 24, 48 and 72 h. **a** Control (untreated) cells showed a normal structure with no remarkable features of apoptosis and necrosis. **b** At 24 h, AO was interconnected with fragmented DNA (*bright green*) and the blebbing cells as an indicator of early apoptosis start to be seen. **c** An *orange colour*, representing late apoptosis, was noticed at 48 h. **d** At 72 h, the cells were orange with a blebbing membrane that indicated late apoptosis. At 72 h, secondary necrotic cells (*bright red colour*) were noticed. **e** The percentages of viable early and late apoptosis and secondary necrotic cells were increased after WEHI-3 cells were treated with BM in a time-dependent manner. Apoptosis increased significantly (*p < 0.05) in a time-dependent manner. VI: viable cells, EA: early apoptosis, LA: late apoptosis, SN: secondary necrosis

### Assessment of the nuclear morphology alterations

In order to confirm the occurrence of apoptosis, cells were treated with Hoechst 33342 stain to observe nuclear condensation; following the treatment with BM, some cells displayed this. However, untreated cells did not show any morphological changes inside their nuclei (Fig. 3).

**Fig. 3:** Effect of BM on nuclear morphological changes of WEHI-3 cells. Control (**a**) and cells treated for 24 h (**b**), 48 h (**c**), and 72 h (**d**), were stained with Hoechst 33,342 after treatment. Apoptotic cells showed a bright blue colour due to DNA condensation; the number increased in a time-dependent manner

### Effect of BM on the ratio of apoptotic cells by Annexin V-FITC staining

The Annexin V-FITC technique was applied to quantify the apoptotic cell population following treatment with BM; after 24 h, the percentage of early apoptotic cells was 17.5%. Continuous exposure of the compound for 48 and 72 h augmented a number of cells undergoing early apoptosis to 23 and 31%, respectively. Meanwhile, the percentage of viable cells after 24 h of treatment was reduced to 73%, compared to 93% of untreated cells. The percentages of cells in late apoptosis and secondary necrosis also significantly increased (*p* < 0.05) in 48 and 72 h, compared to the control cells (Fig. 4).

**Fig. 4:** The influence of BM on inducing apoptosis in WEHI-3 cells. The cells were analysed by flow cytometry after exposure to the treatment in the different times as early or late apoptosis. FITC-conjugated Annexin V and PI were added to each of the control and treated cells. The cells status was presented as healthy (Annexin−/−PI) condensed in the quadrant (Q3–1); early apoptotic (Annexin+/−PI), (Q4–1); late stage of apoptosis (Annexin+/PI+), (Q2–1), where the necrotic cell was (Annexin−/PI+), in (Q1–1). The cell are presented as **a** for control, **b** for 24 h, **c** 48 h, and **d** 72 h. **e** The bar chart presents the percentage of viable and early and late apoptotic cells, showing a significant increase in the number of apoptotic and necrotic cells after BM treatment (*p < 0.05)

### BM elevates the production of the reactive oxygen species

The levels of reactive oxygen species in treating WEHI-3 were rapidly increased at different concentrations of BM (Fig. 5).

**Fig. 5:** Effect of BM on ROS production in the treatment of WEHI-3 cells. After 24 h, 48 h, and 72 h of treatment, DCFH-DA dye was used. The fluorescence then was measured by a microplate reader, p*˂0.05

### Effect of BM on multiparameter cytotoxicity assay on WEHI-3 cells

During the process of cell death, many changes occur in the mitochondria, such as disruption of the mitochondrial membrane potential (MMP); upon this, the transition pores open, with BM showing that there is a significant reduction (*p* < 0.05) in the fluorescence dye after 24 and 48 h of the treatment (Fig. 6). While the cell permeability (CP) was increased in 48 h. The open pores facilitated access to cytochrome C (cytoC) to the cytosol for further apoptosis induction reactions; the release of cytoC was clearly observed at 48 h. Furthermore, the total nuclear intensity (TNI) was increased significantly (*p* < 0.05) at 48 h due to chromatin condensation.

**Fig. 6:** **a** The images of WEHI-3 cells (×20) were treated with BM at IC_50_ for 24 h,48 h and 72 h, stained with different specific dyes, estimating the total nuclear intensity, MMP, cytochrome c release, and cell membrane permeability. **b** The chart quantifies and analyses the apoptosis mediators and parameters of treated WEHI-3 cells. The mediator’s total nuclear intensity (TNI), cell permeability (CP), MMP and cytochrome C (cytoC) showed an elevation in the treated cells, compared to untreated, in a time-dependent manner. The statistically significant differences from untreated cells is expressed as *p < 0.05

### BM increased the activity of caspase 9 and 3

As shown in Fig. 7, BM promoted the enzymatic activity of caspases 9 and 3 significantly in a time-dependent manner (24, 48 and 72 h).

**Fig. 7:** The colorimetric assay was used to determine an activation of caspases 9-and 3/7 in WEHI-3 cells treated by BM in a time-dependent manner; the activities of caspases 9 and 3/7 were increased significantly (*p < 0.05) at different times of treatment

### Effects of BM on the Bcl2 and Bax expression

The apoptotic Bcl2 protein was inhibited by BM at 24, 48 and 72 h. In contrast, the apoptosis-inducer protein, Bax, was up-regulated in the same manner. B-actin protein was used to normalise the results (Fig. 8).

**Fig. 8:** Western blot analysis of the apoptotic and anti-apoptotic protein. **a** Bax, the apoptotic, and Bcl2, the anti-apoptotic proteins, were regulated by BM in 24, 48 and 72h, of the treatment. **b** Quantification of the intensity of bands in ratio to B-actin

### BM arrested the cell cycle at the G1 phase

The cell cycle is a process involved in DNA replication that produces two new identical daughter cells. Normally, it includes five phases: G0 (the resting phase); G1, (the first gap); S (gap for DNA synthesis and replication); G2 (the second gap); and M (mitosis). The disturbance of cell cycle phases caused by BM is presented in Fig. 9. According to the result, BM arrested the WEHI-3 cell cycle at the G0/G1 phase (*p* < 0.05) in a time-dependent manner.

**Fig. 9:** BM has arrested the cell cycle at G0/G1phase. The histograms (**a**) Control, (**b**) 24h, (**c**) 48h, and (**d**) 72h illustrate that G0/G1 is the major phase at which BM could stop the cell cycle, at all times of the treatment. (**e**) Quantification of the different cell phases as G, gap, S, synthesis; M, mitosis

### In vivo anti-leukaemic activity of BM

#### Body, spleen and liver weights

The mean body weight of the leukaemic group was significantly reduced compared to the healthy group (*p* < 0.05). In contrast, the BM treated groups, especially the group receiving the highest dose (60 mg/kg), reached close to the body weight of the vinblastine group. One of the common symptoms of leukaemia is enlargement of the spleen and liver; this was observed in the leukaemic and Tween 20 leukaemic groups when compared to the liver and spleen of normal mice (*p* < 0.05). The 60 mg/kg and vinblastine groups showed a significant reduction in their spleen and liver weights compared to the 30 mg/kg group (Figs. 10 and 11).

**Fig. 10:** The photographs illustrate the spleen and liver of sacrificial mice: BALB/c injected with (1 × 10^6^) WEHI-3 cells (leukaemic mice): and treated groups with 30 mg/kg (*low dose*), 60 mg/kg (*high dose*) of BM, after 3 weeks. The arrows are pointing to the liver (*green arrow*) and spleen (*orange arrow*)

**Fig. 11:** **a** Monitoring of body weight of the different groups for 3 weeks. **b** Spleen weights of all groups (**c**) Liver weights of all groups after 3 weeks

#### Histopathology

The tissue of the spleen simply consists of red pulp to infiltrate the red blood cells, and white pulp to activate the immune response. Six spleens of each mouse group were subjected to histological examination: the leukaemic spleens presented an extension of immature myeloblastic cells into the red pulp. This expansion can be stifled by BM treatments (30, 60 mg/kg), (Fig. 12). The histology of the leukaemic livers showed damaged hepatocytes and distended kupffer cells; this condition improved to normal with healthy hepatocytes with regular nuclei and normal kupffer cells, post-BM treatment (30, 60 mg/kg) (Fig. 13).

**Fig. 12:** Histopathology of the spleen tissues. The image shows (**a**) healthy BALB/c mice with normal white pulp (*green arrow*), red pulp (*blue arrow*) cells plainly visible, contrary to those of the leukaemic mice in whom the white pulp has expanded at the expense of the red pulp areas (**b**, **c**). The histology of the spleen in (**d**) and (**e**) of BM treated groups (30, 60 mg/kg) shows the regression of the white pulp and, at the same time, the red pulp has re-extended; this was also observed in the vinblastine group (**f**)

**Fig. 13:** Histopathology of the liver tissues. The image shows (**a**) normal hepatocytes (*blue arrow*). **b**, **c** BALB/c mice injected with WEHI-3 cells. The leukaemia sectioning shows that the hepatocyte cells were damaged (*blue arrows*), and the kupffer cells are larger (*green arrows*). **d**, **e** BALB/c mice injected with WEHI-3 cells and treated with 30 and 60 mg/kg of BM. **f** Treated by vinblastine: the sections show improvement in the liver histology, compared to the leukaemia groups

#### Detection of apoptosis cells in spleen and liver tissues

The TUNEL assay was used to detect the fragmented chromosome ending of the apoptotic cells in the spleen and liver. In order to evaluate the enhancing effect of BM on apoptosis in vivo*,* six spleens and livers of each mouse group were examined. The dye is bound to DNA and emits a green fluorescence that is visible under a microscope. The green colour was observed at the slides of the spleens and livers of the high dose group (60 mg/kg). However, no apoptotic cells were detected in the spleen and liver of healthy mice (Figs. 14 and 15).

**Fig. 14:** TUNEL assay used to detect the apoptotic cells in spleen tissues. The *yellow arrows* point to an apoptotic cell stained *green*, as shown in the groups treated by BM at 30 mg/kg (**d**), and 60 mg/kg (**e**), and the vinablastine group (**f**). In (**a**) healthy, (**b**) and (**c**) leukaemic groups, no apoptotic cells were detected

**Fig. 15:** TUNEL detection of the apoptotic cells in liver tissues. The *green colour* (*yellow arrows*) indicates the apoptotic cell in the liver of BALB/c mice in (**d**) of the 30 mg/kg, and (**e**) of the 60 mg/kg of BM treated groups, also (**f**) of vinblastine treated mice. **a**, **b** and (**c**) present healthy and leukaemic groups, respectively; clearly, no apoptotic cells were detected

## Discussion

During this a century, highly scientific and commercial attention has been paid to the anticancer properties of natural compounds isolated from plants and herbs in accordance with traditional medicine [16]. Among these compounds are xanthones, which are mostly naturally available in many vegetables and fruits. Several studies have found that xanthones demonstrate anti-inflammatory, antioxidant, antitumor, anti-allergic, antibacterial, antifungal, and antiviral activities [17]. The xanthone molecules alpha and gamma mangostin, which were isolated from the mangosteen fruit, exert anticancer properties; in particular, alpha can reduce prostate malignant hyperplasia [18], whereas gamma can inhibit colon and hepatocellular malignant hyperplasia [19, 20].

The in vitro experiments, as seen in the MTT results, showed that BM had a cytotoxic effect on WEHI-3 cells. Apoptosis is characterised by morphological structure changes, including cell membrane blebbing and DNA segmentation, followed by nucleus breakup and the formation of apoptotic bodies; these signs were observed under the microscopic after staining the treated WEHI-3 cells with AO/PI and Hoechst 33342 to prove the apoptogenic effect of BM in a time-dependent manner in vitro*.*

Throughout apoptosis, the asymmetric distribution of the phospholipid phosphatidylserine (PS), which is a cell membrane constituent located in the inner layer, is predominantly disturbed by translocation to the outer layer [21]. This change in the cell membrane structure is normally recognised by phagocytes that respond by clearing the apoptotic cells from the tissues. PS displays a high affinity to bind selectively with Annexin V in the presence of Ca^2+^ [22]; therefore, this property is used to practically distinguish viable cells from apoptotic cells. Consequently, the current study used this method in the detection of early apoptotic cells using flow cytometry. As a result, shown in Fig. 4, the treated WEHI-3 cells with the IC_50_ concentration of BM prompted the translocation of PS from inner to outer WEHI-3 cell membrane after 24, 48, and 72 h as a result of apoptosis occurrence.

Although reactive oxygen species are a natural by-product in normal cells, its overproduction has a cytotoxic effect and causes disruption in the mitochondrial membrane potential (MMP) and consequently, the mitochondrial apoptosis inducer components such as second mitochondria-derived activator of caspases (SMACs) and (cytoC) were liberated to the cytosol. Released (cytoC) binding with the Apoptotic protease activating factor 1 (Apaf-1) protein to form the apoptosome, which converts procaspase-9 to the active cleaved caspase-9 [23], which in turn activate the procaspase-3 to the cleaved caspase, then stream of reactions stimulate to induce the intrinsic apoptosis pathway [24].

On the other hand, Bcl-2 family has members of proteins involved in anti- apoptosis and apoptosis induction activities to control the intrinsic apoptosis pathway, such as Bcl-2 and Bax. The Bax protein commonly resides in the cytosol, but after receiving the apoptosis signals to the cell, it shifts to associate with the outer mitochondrial membrane, where it forms oligomeric pore with Bak to facilitate the release of (cytoC) and other apoptotic proteins to the cytosol to induce apoptosis reactions [25]. On opposite manner the Bcl-2 protein has an vital role to preserve the cancer cell viability and repress the apoptotic proteins actions such as binding of Bax and Bak which induce the mitochondrial membrane permeabilization, and therefore prevent the release of (cytoC) and ROS to the cytosol to activate the program of the cell death [26]. Immunoblotting techniques were performed to inspect changes in Bax and Bcl-2 expression. As shown in Fig. 8, after cells were exposed to BM at different times, the expression of Bax was up-regulated; however, Bcl-2 expression was down-regulated. These findings indicated that BM could modulate apoptosis by controlling the levels of Bcl-2 and Bax in the WEHI-3 cell line.

Many anticancer drugs work on the mechanism of cell-cycle arrest and/or a combination of both cell-cycle arrest and cell death mechanisms [27]. Considering that the regulation of cell-cycle progression is a potentially powerful strategy for tumour growth control, flow cytometry was used for cell-cycle analysis in this study; our results indicated that BM induced cell-cycle arrest particularly at the G_0_/G_1_ phase in the WEHI-3 cells.

In the in vivo study, the leukaemia symptoms and complications were targeted, such as body, spleen and liver weight and histological changes in the spleen and liver due to disease or treatment. Generally, BM at a low dose (30 mg/Kg) showed a slight improvement in a mouse’s body weight compared to a high dose (60 mg/Kg), which seems to be close to the body weight of the vinablastine positive control group. On the other hand, there is no significant difference in the body weight between the Tween 20 leukaemic group and the leukaemia group.

One of the problems with leukaemia is liver and spleen enlargement, as seen in both the leukaemia and Tween 20 leukaemic groups [28]; therefore, the potency of BM in the treatment of leukaemia is the ability to reduce the weight of the liver and spleen, particularly at a dose of 60 mg/Kg. Deeper investigation of these tissues has been performed using histopathology studies, in which the spleen of leukaemic animals showed an increased accumulation of myloblastic cells covering a large zone, but this extension shrank after the numbers of leukaemic cells were reduced as a result of BM treatment. This inhibited their growth and proliferation and induced apoptosis, and is clearly shown at the dose 60 mg /Kg. This consequence is evidence that BM has a positive influence on improving leukaemia complications. Furthermore, liver histology showed the total tissue damage due to the increased number of neoplastic cells, abnormal hepatocytes and enlarged kupffer cells in the two leukaemic groups (leukaemia and Tween 20 leukaemia);

BM altered this deterioration by lowering the risk of leukaemia on the liver by regressing the numbers of neoplastic cells, minimising the size of the kupffer cells and making the hepatocytes appear healthy, at doses of 30 and 60 mg/Kg.

For confirmation that BM could induce apoptosis, the in vivo TUNEL technique, which detects fragmented DNA in apoptotic cells, was applied to the histological slides of the spleen and liver of all BALB/c mice [29].

No apoptotic cells were detected in the healthy, leukaemia and Tween 20 leukaemic groups, whereas considerable numbers of apoptotic cells were shown in BM-treated groups; these numbers increased with the concentration (60 mg/Kg). These results show that BM fights myelocytic leukaemia in vivo via a stimulated program of cell death.

## Conclusion

We have demonstrated that BM induces apoptosis in WEHI-3 cells, through the intrinsic pathway. The ingestion of BM (at 30 or 60 mg/kg) significantly inhibited WEHI-3 growth in the animal model of leukaemia. Our findings may contribute to a better illustration of the molecular apoptotic mechanisms through which BM exerts its effects on WEHI-3 cells. These results may lead to the development of new chemotherapeutic approaches for the cure of myelomonocytic leukaemia, for which there are no efficient life-prolonging treatments.

## Abbreviations

Bax: Bcl-2–associated X protein
Bcl-2: B-cell lymphoma 2
cytoC: Cytochrome C
DMSO: Dimethylsulphoxide
DNA: Deoxyribonucleic acid
FITC: Fluorescein isothiocyanate
IC_50_: Inhibitory concentration (50%)
MTT: 3-(4,5-Dimethylthiazol-2-yl)-2, 5-diphenyltetrazolium bromide
PBS: Phosphate buffer saline
ROS: Reactive oxygen species
